# Endovascular Repair of the Thoracic Aorta Combined with Drug Therapy in Acute Uncomplicated Type B Aortic Dissection

**DOI:** 10.1155/2022/3021599

**Published:** 2022-09-22

**Authors:** Li Wei, Yan Meng, Guofeng Zhang, Hao Qin

**Affiliations:** ^1^Department of Anesthesiology and Operation, 1st Affiliated Hospital of Xi'an Jiaotong University, Xi'an, China; ^2^Department of Peripheral Vascular Disease, 1st Affiliated Hospital of Xi'an Jiaotong University, Xi'an, China

## Abstract

**Objective:**

This study was to evaluate the clinical efficacy of thoracic endovascular aortic repair (TEVAR) combined with Best Medical Therapy (BMT) in acute uncomplicated type B aortic dissection (TBAD).

**Methods:**

Using the random method, 90 patients admitted to our hospital between January 2018 and January 2020 with acute uncomplicated TBAD were randomly divided into a control group and a study group, with 45 cases in each of the groups. The effectiveness of BMT combined with TEVAR treatment was compared.

**Results:**

The incidence of recent adverse reactions did not differ significantly between the two groups. Compared to the control group, the 1-year survival rate and 2-year survival rate of patients in the study group were considerably higher. In order to examine the relationship between survival and time, the Kaplan-Meier curve was used. Both groups reached the median survival time after 24 months of follow-up. The expected survival time of the study group was longer than that of the control group. False lumen thrombosis or absence of thrombus was significantly more prevalent in the study group than in the control group.

**Conclusion:**

For patients with acute uncomplicated TBAD, BMT combined with TEVAR can significantly improve the long-term survival rate and increase the expected survival time.

## 1. Introduction

Aortic dissection describes the separation of the true and false aortic walls whereby blood from the aortic cavity enters the middle aortic membrane through the tears in the intima of the aorta, which separates the middle membrane and expands along the long axis of the aorta [1]. Acute aortic dissection is a rare and life-threatening condition with a death rate of 1-2% per hour in untreated patients after the onset of symptoms [2].

The symptoms of acute aortic dissection are similar to those of acute myocardial infarction and pulmonary embolism, including severe chest pain, hypotension, or syncope. In addition to the typical symptoms, patients may also experience symptoms of dissection hypoperfusion, such as gastrointestinal discomfort with visceral hypoperfusion, paralysis with spinal hypoperfusion, and lower extremity pain with peripheral hypoperfusion, which can be difficult to diagnose [3, 4].

Stanford's classification method is used to classify aortic dissections into types A and B; TBADs are confined to the abdominal aorta or iliac arteries and can be treated medically, followed by open surgery or endovascular treatment; TBADs can be divided into acute (≤14 days), subacute (14 days~3 months) and chronic (≥3 months) lesions according to their onset date.

The traditional view was that acute TBAD should be operated on as soon as possible in cases of organ ischemia, unrelieved chest pain, and uncontrolled hypertension. Other acute TBAD without complications and stable symptoms may be treated with BMT [5, 6]. The guidelines issued by the American Heart Association and the American College of Cardiology in 2014 listed the drugs that should be adhered to after discharge from acute myocardial infarction, including aspirin enteric-coated tablets, P2Y2 receptor inhibitors, angiotensin-converting enzyme inhibitors/angiotensin II receptor blockers, beta-blockers, and statins that are the best drug therapy for patients with acute myocardial infarction.

Traditional Chinese medicine (TCM), as well as traditional drugs for lowering blood pressure and maintaining heart rate, plays a vital role in the treatment of BMT in TBAD. In TCM, the pathogenesis of TBAD is a result of hyperactivity of the liver Yang and deficiency of the liver and kidney Yin, which primarily manifests through standard manifestations. Chronic pathogenesis is caused by phlegm and blood stasis in the arteries leading to the heart. As defined by the principle of syndrome differentiation, in acute and subacute stages, patients are treated with liver calming Zhengan Xifeng Decoction, which has the functions of nourishing Yang and tonifying the liver and kidney; in chronic stages, patients are treated with Xuefu Zhuyu Decoction, which promotes blood circulation and removes stasis, promotes qi, and relieves pain [7]. In this regard, the treatment of integrated traditional Chinese and Western medicine is a promising research direction in the future.

TEVAR is an innovative minimally invasive technique for implanting stents into the thoracic aorta or thoracoabdominal aorta to treat a wide variety of thoracic aortic lesions; although not suitable for patients' undergoing surgery, it is the preferred treatment due to its lower risk than open thoracic aortic surgery. The surgical success rate of TEVAR in acute or chronic TBAD is 99.1%, and in-hospital mortality rates are 1.6%, with good long-term efficacy [8]. TEVAR has been shown to improve the survival rate in the treatment of uncomplicated Stanford B aortic dissection, but it may still cause complications, and its safety is still in question [9, 10].

In this study, we included patients with acute uncomplicated Stanford type B aortic dissections treated in our hospital with optimal medical therapy and BMT combined with TEVAR. Results are summarized below.

## 2. Data and Methods

### 2.1. General Data

A prospective randomized controlled trial utilizing a single blind design was used for data collection and analysis in this study; we divided 90 patients with type B aortic dissections treated in our hospital between January 2018 and January 2020 into a control group and a study group using a random method, with 45 cases in each group. The randomization was carried out using an online web-based randomization tool (freely available at http://www.randomizer.org/). For concealment of allocation, the randomization procedure and assignment were managed by an independent research assistant who was not involved in screening or evaluation of the participants. The original sample size calculation estimated that 45 patients in each group would be needed to detect a 3-point difference between groups in a 2-sided significance test with a power of 0.8 and an alpha error level of 0.05. Prior to enrollment in this study, the subjects and their family members signed an informed consent form. This study protocol has been approved by the hospital's ethics committee and complies with the ethical guidelines in the Declaration of Helsinki for clinical experiments (registration number: 210237JT/9).

### 2.2. Inclusion and Exclusion Criteria

#### 2.2.1. Inclusion Criteria

1. Patients diagnosed with TBAD male or female over the age of 18
2. Patients with tear distal to the left subclavian artery, without evidence of malperfusion, end-organ ischemia, rupture, or intractable pain
3. Patients who were stable following an acute event
4. Patients who had a contrast-enhanced CT (chest, abdomen, and pelvis) available prior to enrollment

#### 2.2.2. Exclusion Criteria

1. Patients diagnosed with Stanford type A dissection
2. Patients with evidence of Stanford type B dissection
3. Patients diagnosed with traumatic dissection or penetrating ulcer
4. Patients anatomically unsuitable for TEVAR
5. Patients with poor compliance and inability to complete BMT

### 2.3. Methods

#### 2.3.1. BMT

For controlling blood pressure and pain, including, but not limited to, beta-blockers, the following specific methods may be used:

1. Once the patient has been admitted to the hospital, the vital signs, such as blood pressure, electrocardiograms, blood oxygen levels, and other vital signs, are monitored, and the patient must rest.
2. As part of controlling blood pressure, drugs are administered that are aimed at stabilizing systolic blood pressure between 90 mmHg and 110 mmHg in accordance with the principles of perfusion.
3. The administration of drugs that decrease heart rate and inhibit myocardial contractility intravenously. The patient is switched to oral antihypertensive drugs and heart rate-lowering drugs once the clinical symptoms are controlled, and gastrointestinal function has recovered
4. Analgesics should be used rationally for patients experiencing severe pain
5. Dialectically administer the Zhengan Xifeng Decoction and other traditional Chinese medicine treatments

#### 2.3.2. TEVAR

Lidocaine was administered preoperatively to all patients, after which the left radial artery was punctured using the Seldinger approach and a vascular sheath, guide wire, and pigtail catheter were inserted; the angiogram confirmed that the catheter was in the true lumen of the aorta and that the artificial blood vessel pusher was positioned correctly; the sheath should be quickly removed after the blood pressure has been reduced, and the stent graft should be removed; aortic angiography was performed to ensure that the stent was not displaced; once the incision has been closed, the arterial entrance is sutured.

### 2.4. Observational Indicators

Following surgery, all patients were followed up once a month for two years. We evaluated adverse reactions that occurred within the last 30 days, the survival status for all patients during the follow-up period, and the 1-year and 2-year survival rates. To observe the condition of the aortic false lumen, all patients underwent CTA examinations before treatment and at the final follow-up.

### 2.5. Statistical Methods

If the parameter beta is either a difference of means, a log odds ratio, or a log hazard ratio, then it is reasonable to assume that *b* is unbiased and normally distributed. SPSS 23.0 was used to organize and analyze the data in this study; data were checked for normality, and those that did not conform to the normal distribution were converted to normal, expressed as mean ± standard deviation, and a *t*-test was run to determine if there were any statistically significant findings. The enumeration data were expressed as rates, and the chi-square test was used to determine whether there were statistical differences. Survival data were analyzed using Kaplan-Meier, and survival curves were generated using the R software survival package. Significant differences were defined as *α* = 0.05.

## 3. Results

### 3.1. Clinical Data

Table 1 shows that the average age in the control group was 48.13 ± 8.24 years old, with 29 male patients, 18 smokers, 30 hypertensive patients, 5 patients with stroke history, 3 patients with coronary heart disease, and 5 patients with diabetes. In the study group, there were 21 male patients, 15 smoking patients, 19 hypertensive patients, 2 stroke patients, 1 coronary heart disease patient, and two diabetes patients, with an average age of 51.35 ± 10.24. There were no significant differences between the two groups in terms of their basic health status (*P* > 0.05).

### 3.2. Early-Stage Adverse Reactions

As shown in Table 2, there were no cases of endoleak in the control group, four cases of poor perfusion, and three cases of poor perfusion, with a total adverse reaction rate of 13.33% (6/45); in the study group, there were 4 cases of endoleak and 2 cases of poor perfusion, one case and one other case, with a total adverse reaction rate of 20.00% (4/45). A distinct difference in recent adverse reactions did not exist between the two groups (*P* = 0.334).

### 3.3. Comparison of Survival Rates between the Two Groups of Patients

Table 3 shows that, after 1 year of follow-up, 11 patients died in the control group, with a survival rate of 75.56%, and 4 patients died in the study group, with a survival rate of 91.11%; after 2 years of follow-up, 15 patients died in the control group, with a survival rate of 66.67%. In the study group, six patients died, and the survival rate was 86.67 percent. In the study group, survival at one year and survival at two years were significantly greater than those in the control group (*P* < 0.05).

### 3.4. Kaplan-Meier Survival Curves

As shown in Figure 1, Kaplan-Meier curves were used to analyze the relationship between survival and time. In both groups, the median survival period was reached, and the survival rate of the study group was higher by a significant margin in comparison with that of the control group (*P* = 0.024).

### 3.5. CTA Review Results of the Two Groups of Patients

According to Table 4, in the control group, there were 16 cases of false lumen thrombosis or absence of thrombus, 3 cases of false lumen increase, and 11 cases of false lumen no change and 30 cases of false lumen thrombosis, 1 case of false lumen increase, and no change of false lumen in the study group. False lumen thrombosis or absence of thrombus in the study group was significantly higher than that in the control group (*P* = 0.039).

## 4. Discussion

Aortic dissection is a condition when the blood flow of the aorta enters the middle or middle aortic wall from the tear of the intima under the state of high speed and high pressure and continuously expands along the longitudinal axis of the aorta to form a hematoma, separating the media and adventitia of the aorta. In some patients, the adventitia will continue to expand and bulge to form aneurysm. The incidence rate is currently 6/100,000 and is projected to increase year by year, and the age of onset tends to be younger. Aortic dissection can be divided into acute aortic dissection (onset time ≤ 14 d) and chronic aortic dissection (onset time > 14 d) according to the length of onset time. To maintain optimal control of the heart rate and blood pressure, aggressive medical therapy is the gold standard in the treatment of acute uncomplicated TBAD [11, 12]. Recent data suggest, however, that a substantial proportion of patients with acute and uncomplicated TBAD treated with BMT suffer from advanced aortic-related complications, such as aneurysmal degeneration, which can increase mortality and require reiterative intervention [13]. An alternative to open surgery, TEVAR offers a shorter hospital stay and a faster recovery time than traditional open procedures for repairing thoracic aortic aneurysms or dissections [14, 15]. This study involved the use of BMT combined with TEVAR in the study group. The results showed that there was no significant difference in the rate of early complications between the two groups. The 1-year survival rate and 2-year survival rate of the study group were significantly greater than those of the control group. The possible explanation is that TEVAR used stent-graft to cover the proximal breach to induce false lumen thrombosis, increase blood perfusion in the true lumen, improve blood supply to distal organs, and ultimately promote aortic remodeling. Although the torn intimal sheet in patients with acute aortic dissection involving the common iliac artery at the distal end is likely to involve the renal artery orifice or affect the renal artery blood supply due to renal artery dissection, TEVAR treatment can improve true lumen perfusion and distal visceral blood supply, and the expected survival time was significantly longer than that of the control group. As a result, the incidence of false lumen thrombosis or disappearance in the study group was significantly higher than that in the control group.

BMT is performed in order to reduce aortic wall stress and false lumen pressure, and intravenous drugs are administered in the acute phase in order to control heart rate and blood pressure, as well as to reduce the maximum change in left ventricular pressure during early systole (maximum dP/dt) [16]. The use of intravenous beta-blockers is the first line of therapy for reducing blood pressure and dP/dt. Whenever a potent vasodilator, such as sodium nitroprusside, is to be used, it must be ensured that the patient is also taking a beta-blocker with good rate control to prevent reflex tachycardia [17]. In addition, appropriate analgesia should be given to control pain and prevent the activation of the sympathetic nervous system, which may lead to tachycardia and poor control of blood pressure [18]. Generally, the heart rate should not exceed 70 beats per minute, and the systolic blood pressure should not exceed 120 millimeters of mercury. In the event that the patient's blood pressure and heart rate are controlled and they are able to tolerate an oral diet, antihypertensive therapy can be switched to an oral regimen that will last for life. BMT is essential for all TBAD patients, but patient compliance is low, which limits its efficacy.

In TEVAR, endoleaks are the most common complication, caused by the failure to completely isolate the communication between the aneurysm cavity and arterial blood flow after stent release for aortic dissection [19]. A common complication of TBAD is malperfusion syndrome, which is caused by static or dynamic occlusion of branch vessels in the affected aortic segment. The incidence of endoleak after TEVAR in this study was 8.89%, and the total complications were not statistically different from those associated with BMT. TEVAR for acute TBAD without problems is controversial; however, it did not result in an increase in early complications in this research. Furthermore, the 2022 American College of Thoracic Surgeons/American Society of Thoracic Surgeons clinical recommendations for type B aortic dissection said that preventive TEVAR might be explored in patients with simple TBAD to minimize late aortic-related events and aortic-related fatalities [20]. The evidence level is B, which also enables TEVAR implementation. The enhanced TEVAR surgical techniques and stents are among the reasons why it is preferable than BMT alone. In previous studies, the time span was long, and the surgical procedure was different, which may affect the long-term outcome [21].

This study believes that the aorta of the descending thoracic aorta is remodeled well, because the stent-graft seals the first rupture of the dissection, the true lumen increases under the radial support force of the stent-graft, and the false lumen cannot penetrate the first rupture. Or other breaks in the descending thoracic aorta to obtain blood flow and blood stasis occurs, resulting in the formation of thrombus and the final organic absorption [22]. Collectively, no significant changes in distal false lumen diameter and total aortic diameter during TEVAR follow-up suggest that dissection may be stable, and short-term distal ruptures do not require surgical treatment, but strict imaging follow-up is very important for patients with untreated distal ruptures [23, 24]. Long-term follow-up studies are needed to provide answers on whether and how to treat distal ruptures in the long term. This study provides certain therapeutic ideas for the future clinical treatment of acute aortic dissection. However, this study is a single-center study with a small sample size. In addition, because the center has not yet carried out emergency coronary artery bypass surgery, these patients were not included in the study. The results and conclusions obtained still need to be further confirmed by multicenter and large-sample studies.

## 5. Conclusion

In conclusion, for patients with acute uncomplicated TBAD, BMT combined with TEVAR can improve the long-term survival rate, increase the predicted survival time, and is generally safe. Although this study did not use animal experiments or in vitro and in vivo experiments to study the mechanism, it also provided a certain research direction for future basic experiments and a certain choice for early clinical treatment, paving a way for future protein model simulation and drug design.

## Figures and Tables

**Figure 1:** Kaplan-Meier analysis of survival status.

**Table 1:** Comparison of general data.

	Control group	Study group	*t*/*χ*^2^	*P*
*n*	45	45		
Age	48.13 ± 8.24	51.35 ± 10.24	0.164	0.104
Gender (male/female)	29/16	31/14	0.200	0.655
Smoking	18	15	0.431	0.512
Background disease			0.710	0.871
Hypertension	30	19		
Stroke	5	2		
CHD	3	1		
Diabetes	5	2		

**Table 2:** Early-stage adverse reactions.

	Endoleak	Poor perfusion	Others	Total
Control group (*n* = 45)	0	4	2	6 (13.33%)
Study group (*n* = 45)	4	2	3	9 (20.00%)
*χ* ^2^				0.720
*P*				0.396

**Table 3:** Comparison of survival rates between the 2 groups of patients (*n*, %).

	1-year survival rate	2-year survival rate
Control group (*n* = 45)	34 (75.56%)	30 (66.67%)
Study group (*n* = 45)	41 (91.11%)	39 (86.67%)
*χ* ^2^	3.920	5.031
*P*	0.048	0.025

**Table 4:** CTA review results of the two groups of patients.

	Thrombus or absence of thrombus	Increase	No change
Control group (*n* = 30)	16	3	11
Study group (*n* = 39)	30	1	8
*χ* ^2^	4.246	1.717	2.217
*P*	0.039	0.190	0.136

## Data Availability

All data generated or analyzed during this study are included in this published article.
